The article "Long noncoding RNA CASC9 promotes the proliferation and metastasis of papillary thyroid cancer via sponging miR‐488‐3p" was retracted in 2024. Reasons: manipulated images; plagiarized images; duplicated images; overlap with other authors' work.

# Long noncoding RNA CASC9 promotes the proliferation and metastasis of papillary thyroid cancer via sponging miR‐488‐3p

**DOI:** 10.1002/cam4.2839

**Published:** 2020-01-13

**Authors:** Yonghui Chen, Yaomei Li, Hongbo Gao

**Affiliations:** ^1^ Department of Nuclear Medicine Peking Union Medical College Hospital Chinese Academy of Medical Sciences and Peking Union Medical College Beijing China; ^2^ Beijing Key Laboratory of Molecular Targeted Diagnosis and Therapy in Nuclear Medicine Beijing China; ^3^ Department of Nuclear Medicine The Mine Hospital of Xuzhou Xuzhou China; ^4^ Department of Radionuclide Treatment Center Beijing Nuclear Industry Hospital Beijing China

**Keywords:** long noncoding RNA CASC9, metastasis, miR‐488‐3p/ADAM9, papillary thyroid cancer, proliferation

## Abstract

Cancer susceptibility candidate 9 (CASC9) is a recently identified lncRNA that acted as a tumor promotor in diversified cancer types. However, its role in papillary thyroid cancer (PTC) remains unknown. The expression of CASC9 was measured in 52 human PTC tissues and PTC cell lines as well as their controls. The proliferation, migration, and invasion of PTC cells were determined after knockdown or overexpression of CASC9 to evaluate the effect of CASC9 on PTC cells. Also, the role of PTC tumorigenesis was confirmed in mice xenograft models. Additionally, the underlying mechanisms of CASC9 were further researched. We found that CASC9 expression was augmented in human PTC tissues and cells. Higher CASC9 expression was associated with large tumor size, advanced stage, or lymph node metastasis. Downregulation of CASC9 significantly attenuated the proliferative, migrative, and invasive abilities of PTC cells, and suppressed tumorigenesis in vivo. While overexpression of CASC9 elevated the proliferation, migration, and invasion of PTC cells. miR‐488‐3p expression was decreased, and ADAM9 level was increased in PTC tissues and cells. CASC9 expression was negatively related to miR‐488‐3p, but positively associated with ADAM9 expression in PTC tissues. Molecular mechanism analysis revealed that CASC9 functioned via sponging miR‐488‐3p to regulate ADAM9 expression, followed by activation of EGFR‐Akt signaling. In conclusion, lncRNA CASC9 promoted the malignant phenotypes of PTC via modulating miR‐488‐3p/ADAM9 pathway. This study may provide a novel therapeutic target for the treatment of PTC.

## 1 INTRODUCTION

Thyroid cancer is the most frequent endocrine malignancy. Its incidence is increasing all over the world. About 567 000 new cases were reported worldwide both in men and women in 2018.^1^ Thyroid cancer mostly occurs in women and the global incidence in women is three times higher than in men.^1^ Although the diagnosis and treatment approaches have improved greatly, mortality rates from thyroid cancer have changed minimally.^1^, ^2^ Papillary thyroid cancer (PTC) is the major subtype of this cancer, accounting for over 80% of all thyroid cancer.^3^, ^4^ Patients with PTC carried a relatively favorable prognosis; however, a certain part of PTC patients suffered from metastasis to lymph nodes and lungs, leading to the poor clinical outcomes.^2^, ^5^, ^6^, ^7^ Studies have demonstrated that genetic and epigenetic alterations play important roles in the development of PTC.^8^, ^9^ However, the underlying molecular mechanisms remain poorly characterized. Therefore, clarifying the mechanisms associated with the pathogenesis of PTC may help to improve the therapeutic strategies for this cancer.

Long noncoding RNAs (lncRNAs) are one important member of noncoding RNAs. They are longer than 200 nucleotides that have limited protein‐coding functions. Accumulating evidences indicated that lncRNAs display diverse roles in modulating gene transcription, posttranscription, translation, and epigenetic regulation.^10^, ^11^ LncRNAs are abnormally expressed or dysregulated to mediate multiple human diseases, including cancers.^11^, ^12^, ^13^, ^14^ LncRNAs have been demonstrated to participate in the development of PTC. For example, lncRNA ABHD11‐AS1 was elevated in PTC, and it augmented the proliferation, migration, and invasion, and suppressed apoptosis of PTC cells by miR‐199a‐5p/SLC1A5 axis.^15^ The expression of lncRNA AB074169 was decreased in PTC, and overexpression of AB074169 caused cell cycle arrest and inhibited tumor growth.^16^ LncRNA AB074169 acted as a tumor suppressor in PTC via modulating KHSRP‐mediated CDKN1a expression.^16^

Cancer susceptibility candidate 9 (CASC9) is located on human chromosome 8q21.11.^17^ It was originally identified as a lncRNA related to esophageal squamous cell carcinoma (ESCC).^17^ CASC9 expression was increased in ESCC clinical samples and cells. Downregulation of CASC9 inhibited migration and invasion of ESCC cells.^17^ Subsequently, the roles of CASC9 in other cancer types were demonstrated. Studies have found that CASC9 expression was elevated in breast cancer,^18^ colorectal cancer,^19^ oral squamous cell carcinoma,^20^ ovarian cancer,^21^ lung adenocarcinoma,^22^ gastric cancer,^23^ and glioma,^24^ and CASC9 functioned as a tumor promotor in these cancers. However, the expression pattern and role of CASC9 in PTC remain unrevealed. In the current study, the expression of CASC9 was examined in human PTC tissues and cell lines. Additionally, the role and mechanism of CASC9 in PTC were investigated by loss‐of‐function assays both in vitro and in xenograft mice models.

## 2 MATERIALS AND METHODS

### 2.1 Human tissue collection

A total of 52 pairs of PTC and adjacent normal thyroid tissues (>3 cm from tumor borders) were obtained from patients who underwent thyroidectomies at Peking Union Medical College Hospital and The Mine Hospital of Xuzhou, from December 2016 to May 2018. All patients did not receive any local or systemic treatments before surgery. After confirming by two pathologists independently, collected fresh tissue samples were frozen in liquid nitrogen. All patients enrolled signed informed consent. This experiment was approved by the Research Ethics Committee of Peking Union Medical College Hospital.

### 2.2 Cell culture and transfection

Normal human thyroid cell line, Nthy‐ori3‐1, and two human PTC cell lines (TPC‐1 and BCPAP) were used in this study and they were purchased from Shanghai Huiying biological technology co., Ltd. TPC‐1 and Nthy‐ori3‐1 cells were cultured in RPMI‐1640 medium, and BCPAP cells were maintained in Dulbecco's Modified Eagle's medium. Both cell culture medium contains 10% fetal bovine serum (FBS) and 1% penicillin/streptomycin. These cells were grown in a cell incubator with 5% CO_2_ at 37°C.

The CASC9 interfering plasmid pLVX‐CASC9‐short hairpin RNA (CASC9 shRNA) was constructed (Target sequence 5'‐GCCCAGAAGACAGTGGAATGA‐3') to downregulate CASC9 expression. And, a scrambled sequence was inserted into pLVX‐shRNA1 plasmid, which was used as the control. CASC9 and ADAM9 overexpression plasmid pcDNA3.1‐CASC9 and pcDNA3.1‐ADAM9 were used to upregulate CASC9 and ADAM9 expression, respectively. miR‐488‐3p mimic, miR‐488‐3p antagomir (anti‐miR‐488‐3p), and their controls were purchased from GenePharma. Both PTC cell lines were transfected with the above vectors using Lipofectamine 3000 reagent (Invitrogen) following the manufacturer's instructions.

### 2.3 Cell proliferation analysis

The proliferation of TPC‐1 and BCPAP cells was analyzed by Cell counting kit‐8 (CCK‐8; Beyotime). Briefly, these cells were transfected with designated vectors for 24 hours and then reseeded into 96‐well plates at a density of 4 × 10^3^ cells/well (a total of 100 μL). Cell proliferation ability was evaluated at different time points (0, 24, 48, and 72 hours) after planting by adding 10‐μL CCK‐8 solution. After culturing at 37°C for 30 minutes, a Microplate Reader (Bio‐Rad) was used to determine the absorbance at 450 nm.

### 2.4 Wound healing assay

Transfected PTC cells were seeded into 6‐well plates at 3 × 10^5^ cells/well until approximately 90% confluent. A scratch was made using a 200‐µL sterile pipette tip, and phosphate buffered saline (PBS) was used to wash the cells. Subsequently, cells were cultured in serum‐free medium for another 24 hours, the widths of the scratches were imaged under a microscope, and calculated using ImageJ software.

### 2.5 Transwell assay for cell invasion

After 24 hours transfection, 24‐well Transwell chambers (8‐μm pores; Millipore) with Matrigel (BD) were utilized to perform transwell invasion assay. TPC‐1 and BCPAP cells, which were in serum‐free medium, were planted in the apical chamber. The basolateral chamber was imbued with 600‐μL culture medium containing 20% FBS. These cells were maintained at 37°C for another 24 hours. Cells, which did not traverse the filter, were wiped off using a cotton swab, and cells on the underside of the membrane were fixed with 4% formaldehyde, stained with 0.1% crystal violet, and photographed with a light microscope. The experiments were carried out independently in triplicate.

### 2.6 Bioinformatic analysis and dual‐luciferase reporter assay

Bioinformatic analysis using Starbase showed that both CASC9 and ADAM9 possess the binding sites of miR‐488‐3p. CASC9 cDNA was amplified from human PTC tissues and inserted into pGL3 plasmid. Also, the mutant miR‐488‐3p‐binding sequence was introduced to construct the CASC9 mutant plasmid. TPC‐1 cells were seeded into 48‐well plates, followed by incubation for 24 hours. Then, cells were transfected with CASC9‐WT or CASC9‐MUT plasmid in combination with miR‐488‐3p/control mimic using Lipofectamine 3000. After transfection for 48 hours, the relative luciferase activity of each well was analyzed by a Dual‐Luciferase Assay Kit (Promega).

### 2.7 RNA immunoprecipitation assay

In BCPAP cells, an RNA immunoprecipitation (RIP) assay was developed using an EZ‐Magna RIP RNA‐Binding Protein Immunoprecipitation Kit (Millipore) with anti‐human Ago2 antibody as previously described.^25^ The precipitated RNAs were isolated to determine the expression of CASC9 and ADAM9 using real‐time PCR analysis.

### 2.8 Mouse xenograft model

Twelve female BALB/c nude mice (5‐ to 6‐week‐old) were obtained from Beijing Vital River Laboratory Animal Technology Co., Ltd and housed under specific pathogen‐free conditions. All animal procedures were approved by the Animal Care Committee of Peking Union Medical College Hospital. Mice were randomly divided into two groups, and each group contains six mice. For xenograft models, 1 × 10^7^ BCPAP cells stably transfected with CASC9 shRNA or negative control were subcutaneously injected into the back flanks of mice. The tumor volume was determined every 5 days using the following formula: (Length × Width^2^)/2. All mice were executed 30 days after implantation. Tumors were collected for further study.

### 2.9 Real‐time PCR

Trizol reagent (Invitrogen) was used to extract total RNAs from tissues and cultured cells. To analyze the expression of CASC9 and ADAM9, 2‐μg total RNA was used for reverse transcription reaction by M‐MLV Reverse Transcriptase (Promega), followed by Real‐time PCR analysis with SYBR Green Real‐time Master Mix (Toyobo). CASC9 and ADAM9 expression levels were measured using the 2^−ΔΔCt^ method normalized to GAPDH. To detect miR‐488‐3p expression, TaqMan MiRNA Reverse Transcription Kit and TaqMan Human MiRNA Assay Kit (Applied Biosystems) were used as the instructions. miR‐488‐3p expression was measured with normalization to U6 snRNA.

### 2.10 Western blot

Proteins were extracted from tissues and cells with RIPA lysis buffer (Beyotime) including cocktail, a protease inhibitor. Protein concentrations were examined by a protein assay kit (Bio‐Rad). Thirty microgram of protein was separated by SDS‐PAGE. After that, the protein was electroblotted onto PVDF membranes (Millipore). The membrane was immunoblotted with primary antibodies against ADAM9, epidermal growth factor receptor (EGFR), p‐EGFR, Akt, p‐Akt, and GAPDH (both from Abcam) overnight at 4°C. After washing with PBS‐Tween 20 (PBST), the membrane was incubated with HRP‐labeled secondary antibody for 1 hour. Signals were developed with ECL detection reagent (Thermo Fisher). The relative expression level of ADAM9 was calculated by ImageJ software with normalization to GAPDH.

### 2.11 Statistical analysis

All in vitro experiments were performed in triplicates independently. Results are presented as mean ± SD. Statistical analyses between groups were performed by Student's *t* test or Mann‐Whitney *U* test. Differences more than two groups were analyzed by one‐way ANOVA followed by Bonferroni post hoc test. Chi‐squared test was used to assay the relationship between CASC9 and patients’ clinicopathological characteristics. The correlation between CASC9 and miR‐488‐3p or ADAM9 in PTC tissues was measured by Pearson's correlation analysis. Data analysis was handled with SPSS19.0 software. Values were considered significant at *P* < .05.

## 3 RESULTS

### 3.1 CASC9 expression is elevated in PTC tissues and cell lines

We firstly measured the expression of CASC9 in 52 PTC tissues by real‐time PCR. The results showed that CASC9 expression was higher in PTC tissues than that in adjacent normal thyroid tissues (Figure 1A). The involvement between CASC9 and clinicopathological parameters was further analyzed. We found that higher CASC9 expression was related to large tumor size, advanced stage, or lymph node metastasis. No significant correlation was noted between CASC9 expression and other clinical features, including age, gender, or multifocality (Table 1). Then, CASC9 expression was detected in two human PTC cell lines. As shown in Figure 1B, CASC9 expression was higher in TPC‐1 and BCPAP PTC cells than that in normal human thyroid Nthy‐ori3‐1 cells.

**Figure 1:** Cancer susceptibility candidate 9 (CASC9) expression was elevated in papillary thyroid cancer (PTC) tissues and cell lines. (A) The expression of CASC9 in 52 PTC tissues and adjacent normal tissues was analyzed by real‐time PCR. B, CASC9 level in normal human thyroid cell line Nthy‐ori3‐1 and two human PTC cell lines (TPC‐1 and BCPAP). *P < .05 vs the normal group or Nthy‐ori3‐1 cells

**Table 1:** Correlation between Cancer susceptibility candidate 9 (CASC9) expression and clinicopathological characteristics of 52 PTC patients

Characteristics	Number	CASC9 expression		*P*
		Low (n = 26)	High (n = 26)	
Age				
<45	31	18	13	.158
≥45	21	8	13	
Gender				
Male	17	7	10	.375
Female	35	19	16	
Tumor size				
<2 cm	23	16	7	.012*
≥2 cm	29	10	19	
Multifocality				
Present	27	12	15	.405
Absent	25	14	11	
Lymph node metastasis				
Negative	22	16	6	.005*
Positive	30	10	20	
TNM stage				
I/II	33	21	12	.01*
III/IV	19	5	14	

Note

Chi‐squared test.

TNM, Tumor Node Metastasis

* *P* < .05.

### 3.2 CASC9 promotes the proliferation, migration, and invasion of PTC cells

The role of CASC9 in PTC was analyzed by downregulation or overexpression of CASC9. As shown in Figure 2A, the CASC9 shRNA notably decreased CASC9 expression, whereas pcDNA3.1‐CASC9 significantly elevated CASC9 expression. CCK‐8 analysis displayed that knockdown of CASC9 reduced the proliferation of TPC‐1 and BCPAP cells (Figure 2B). The migratory abilities of PTC cells were suppressed after downregulation of CASC9, which was revealed by a wounding healing assay (Figure 2C). Transwell assay was conducted to measure the influence of CASC9 on the invasion of PTC cells. Results demonstrated that compared with cells transfected with control shRNA, the number of invasive cells transfected with CASC9 shRNA was decreased (Figure 2D). The results also showed that overexpression of CASC9 facilitated the proliferation, migration, and invasion of TPC‐1 and BCPAP cells (Figure 2B‐D). Herein, the data indicated that CASC9 could promote the proliferation, migration, and invasion of PTC cells.

**Figure 2:** Cancer susceptibility candidate 9 (CASC9) promotes the proliferation, migration, and invasion of papillary thyroid cancer cells. A, CASC9 expression was reduced in TPC‐1 and BCPAP cells transfected with sh‐CASC9, but increased in cells transfected with pcDNA3.1‐CASC9. B, TPC‐1 and BCPAP cells were transfected with sh‐NC/sh‐CASC9 or pcDNA3.1/pcDNA3.1‐CASC9, cell viability was analyzed by CCK‐8 assay. C, The migratory abilities of TPC‐1 and BCPAP cells were determined using wounding healing assay. D, Transwell analysis for the invasion of TPC‐1 and BCPAP cells. *P < .05 vs the sh‐NC group, ^#^ *P* < .05 vs the pcDNA3.1 group

### 3.3 CASC9 directly binds to and modulates miR‐488‐3p in PTC cells

Next, the mechanism of CASC9 was determined. The target prediction tool Starbase showed that CASC9 has the potential binding sites for miR‐488‐3p. The putative binding sequence was revealed in Figure 3A. Their relationship was further confirmed and we found that miR‐488‐3p mimic dramatically suppressed the luciferase activity of CASC9‐WT, but not the luciferase activity of CASC9‐MUT compared to the control mimic (Figure 3B). We also found that miR‐488‐3p expression was remarkably enhanced in TPC‐1 and BCPAP cells with CASC9 knockdown (Figure 3C). Moreover, miR‐488‐3p expression was decreased in human PTC tissues compared to matched para‐cancerous tissues (Figure 3D). Importantly, we found that a negative relationship existed between CASC9 and miR‐488‐3p in tumor tissues (Figure 3E). Also, miR‐488‐3p expression was decreased in PTC cells compared with Nthy‐ori3‐1 cells (Figure 3F). These results indicated that CASC9 may function by sponging miR‐488‐3p.

**Figure 3:** Cancer susceptibility candidate 9 (CASC9) directly binds to and regulates miR‐488‐3p in papillary thyroid cancer (PTC). A, The binding sites of CASC9 and ADAM9 with miR‐488‐3p. B, miR‐488‐3p mimic suppressed the luciferase activity of CASC9 wild‐type vector in TPC‐1 cells. C, TPC‐1 and BCPAP cells were transfected with sh‐NC or sh‐CASC9, and miR‐488‐3p expression was detected by real‐time PCR. D, The expression of miR‐488‐3p was decreased in 52 PTC tissues compared with that in adjacent normal tissues. E, Pearson's correlation analysis for the correlation between CASC9 and miR‐488‐3p in 52 PTC tissues. F, miR‐488‐3p expression in Nthy‐ori3‐1 normal thyroid cells and PTC cells. *P < .05 vs the NC mimic group, ^#^ *P* < .05 vs the sh‐NC group, ^&^ *P* < .05 vs the normal group or Nthy‐ori3‐1 cells

### 3.4 CASC9 functions via mediating miR‐488‐3p in PTC cells

The role of miR‐488‐3p in PTC cells was analyzed. As shown in Figure 4, miR‐488‐3p mimic inhibited the proliferation, migration, and invasion of TPC‐1 and BCPAP cells. Contrarily, anti‐miR‐488‐3p promoted these features of PTC cells (Figure 4). These data indicated that miR‐488‐3p could attenuate the proliferation, migration, and invasion of PTC cells.

**Figure 4:** miR‐488‐3p inhibits the proliferation, migration, and invasion of papillary thyroid cancer cells. TPC‐1 and BCPAP cells were transfected with miR‐488‐3p mimic, anti‐miR‐488‐3p, or their controls. A, Cell viability was examined by CCK‐8. B, The migration of cells was measured by wounding healing assay. C, Cell invasion ability was detected by transwell. *P < .05 vs the NC mimic group, ^#^ *P* < .05 vs the anti‐NC group

We further investigated whether CASC9 functions via mediating miR‐488‐3p. The results demonstrated that the effects of CASC9 silencing on the proliferation, migration, and invasion of TPC‐1 and BCPAP cells were abrogated by anti‐miR‐488‐3p. However, miR‐488‐3p mimic further strengthened the effect of CASC9 downregulation (Figure 5). In summary, these results suggested that CASC9 facilitated the proliferation, migration, and invasion of PTC cells by negatively regulating miR‐488‐3p in PTC cells.

**Figure 5:** Cancer susceptibility candidate 9 (CASC9) functions via negatively regulating miR‐488‐3p. TPC‐1 and BCPAP cells were transfected with sh‐CASC9 and miR‐488‐3p mimic/anti‐miR‐488‐3p or transfected with sh‐NC/sh‐CASC9 only. A, CCK‐8 was used to assay cell viability. B, Wounding healing analysis for cell migration. C, The invasion of these cells under different treatment was determined by transwell. *P < .05 vs the sh‐NC group, ^#^ *P* < .05 vs the sh‐CASC9 group

### 3.5 CASC9 regulates ADAM9‐EGFR‐Akt signaling by sponging miR‐488‐3p

This study has shown that miR‐488‐3p could regulate ADAM9 expression.^26^ ADAM9 has been found to be responsible for the migration and invasion of thyroid cancer.^27^ Hence, we further verified the relationship between CASC9 and ADAM9 in PTC. ADAM9 expression was higher in PTC tissues and cells than their controls (Figure 6A,B). There was a positive association between CASC9 and ADAM9 in PTC samples (Figure 6C). An RIP assay with anti‐Ago2 antibody revealed that the enrichment of Ago2 on CASC9 was decreased, but enrichment on ADAM9 was elevated after CASC9 downregulation (Figure 6D). Furthermore, miR‐488‐3p mimic notably decreased ADAM9 expression both in TPC‐1 and BCPAP cells. Knockdown of CASC9 reduced ADAM9 expression, which was attenuated by anti‐miR‐488‐3p, but further strengthened by miR‐488‐3p mimic (Figure 6E,F). Also, both CASC9 knockdown and miR‐488‐3p mimic could suppress the activation of EGFR and Akt, as demonstrated by deceased phosphorylation of EGFR and Akt. The influences of CASC9 shRNA on the activation of EGFR and Akt were restored by anti‐miR‐488‐3p, whereas enhanced by miR‐488‐3p mimic (Figure 6F). In addition, the suppressed proliferation, migration, and invasion of PTC cells by CASC9 silencing were attenuated by ADAM9 upregulation (Figure 6G‐I). These results demonstrated that CASC9 functioned in PTC cells via regulating ADAM9 expression by sponging miR‐488‐3p.

**Figure 6:** Cancer susceptibility candidate 9 (CASC9) regulates ADAM9 expression by sponging miR‐488‐3p in papillary thyroid cancer (PTC). A, ADAM9 expression was detected by real‐time PCR in 52 human PTC tissues and adjacent normal tissues. B, ADAM9 expression was determined in Nthy‐ori3‐1, TPC‐1, and BCPAP cells. C, The correlation between ADAM9 and CASC9 in 52 PTC tissues. D, BCPAP cells were transfected with sh‐NC or sh‐CASC9 for 72 h, an RIP assay with anti‐Ago2 antibody was performed, and the levels of CASC9 and ADAM9 enrichment on Ago2 were analyzed. E, The mRNA levels of ADAM9 were detected in TPC‐1 and BCPAP cells under different treatments. F, Protein levels of ADAM9, p‐EGFR, EGFR, p‐Akt, and Akt in TPC‐1 and BCPAP cells were determined by western blot. G, PTC cells were transfected with sh‐CASC9 with or without ADAM9, cell viability was determined by CCK‐8. H, The migration of TPC‐1 and BCPAP cells was measured by wounding healing analysis. I, transwell assay for the invasion of TPC‐1 and BCPAP cells. *P < .05 vs the normal group, Nthy‐ori3‐1 cells, or NC mimic group, ^#^ *P* < .05 vs the sh‐NC group, ^&^ *P* < .05 vs the sh‐CASC9 group

### 3.6 CASC9 downregulation decreases tumor growth in vivo that is related to miR‐488‐3p/ADAM9 axis

The effect of CASC9 on PTC was validated in xenograft mouse models. CASC9 shRNA significantly reduced CASC9 expression in mice tumor tissues (Figure 7A). Tumor volume was notably reduced in the CASC9 shRNA group compared to the control (Figure 7B). As excepted, downregulation of CASC9 significantly reduced tumor weight (Figure 7C). The expression of miR‐488‐3p was elevated, while ADAM9 level was decreased in tumor tissues from mice transfected with CASC9 shRNA compared with the control shRNA (Figure 7D,E). These data indicated that CASC9 knockdown decreased tumor growth in mice, which was associated with miR‐488‐3p/ADAM9 pathway.

**Figure 7:** Cancer susceptibility candidate 9 (CASC9) downregulation decreases tumor growth in vivo through miR‐488‐3p/ADAM9 axis. BCPAP cells stably transfected with CASC9 shRNA or negative control were subcutaneously injected into the back flanks of BALB/c nude mice. Mice were sacrificed 30 d after implantation. A, CASC9 expression in tumor tissues was analyzed by real‐time PCR. B, Tumor volume was determined every 5 d after injection. C, Tumor weight was measured after sacrificed. The expression of miR‐488‐3p (D) and ADAM9 (E) was detected in mice tumor tissues. N = 6 per group. *P < .05 vs the sh‐NC group

## 4 DISCUSSION

Increasing studies have shown that lncRNAs participate in the initiation and progression of cancers, including PTC.^11^, ^28^, ^29^ In this study, we found that CASC9 expression was elevated in human PTC tissues and cells. It facilitated the proliferation and metastasis of PTC via modulating miR‐488‐3p/ADAM9/EGFR‐Akt axis.

In recent years, the studies of CASC9 are drawing more and more attention in cancers. Wu et al^30^ showed that CASC9 expression was increased in ESCC tissues. Its expression was positively involved in tumor size and TNM stage, and its high level predicted poor overall survival of patients with ESCC. Interfering CASC9 suppressed ESCC cell growth and blocked cell cycle G1/S transition in vitro, as well as inhibited tumorigenesis in nude mice.^30^ It functioned via suppressing PDCD4 expression by recruiting enhancer of zeste homolog 2 and subsequently altering H3K27me3 level in PDCD4 promoter.^30^ CASC9 also facilitated ESCC metastasis via elevating LAMC2 expression by regulating CREB‐binding protein‐mediated histone acetylation.^31^ The expression of CASC9 was increased in ovarian cancer tissues and cells and an enhanced level predicted an unfavorable prognosis in ovarian cancer patients. CASC9 accelerated ovarian cancer cell proliferation, invasion, and migration via acting as a competing endogenous RNA (ceRNA) for miR‐758‐3p to modulate LIN7A expression.^21^ CASC9 enhanced breast cancer cell proliferation and metastasis through positively regulating CHK1 via sponging the miR‑195/497 cluster 32 or through miR‐215/TWIST2 signaling.^18^ Elevated CASC9 promoted oral squamous cell carcinoma progression by inhibiting autophagy‐mediated apoptosis.^20^ However, the influence of CASC9 in PTC remains enigmatic. Hence, this study investigated the role of CASC9 in PTC. We found that CASC9 expression was higher in PTC tissues than in adjacent normal tissues. Elevated CASC9 level was associated with poor clinicopathological features. Also, CASC9 expression was boosted in PTC cells. This suggested that CASC9 may be a regulator in PTC. Our further study demonstrated that knockdown of CASC9 suppressed the proliferation, migration, and invasion of PTC cells in vitro, and inhibited tumor growth in vivo. Whereas CASC9 overexpression elevated the proliferation, migration, and invasion of PTC cells. These results indicated that CASC9 could promote the proliferation and metastasis of PTC.

LncRNAs participate in various biological process mainly via acting as ceRNAs.^33^ The mechanism of CASC9 in PTC was mainly focused on the ceRNA regulation. miR‐488‐3p was found to be an important tumor suppressor in various cancers.^34^, ^35^ In this study, we found that miR‐488‐3p expression was decreased in PTC tissues and cells. miR‐488‐3p mimic suppressed, whereas anti‐miR‐488‐3p promoted the proliferation, migration, and invasion of PTC cells, which demonstrated that miR‐488‐3p played tumor‐suppressing roles in PTC. Next, we further investigated the relationship between CASC9 and miR‐488‐3p. Bioinformatic analysis showed that CASC9 has the putative binding sites for miR‐488‐3p, and dual‐luciferase reporter assay verified their direct combination. And, CASC9 could negatively regulate miR‐488‐3p expression in PTC cells. As expected, miR‐488‐3p expression was negatively related to CASC9 in PTC tissues. In addition, anti‐miR‐488‐3p significantly reversed the suppressed proliferation, migration, and invasion of PTC cells by CASC9 downregulation. And, miR‐488‐3p mimic further strengthened the effects of CASC9 silencing on PTC cells. In general, these data suggested that CASC9 functioned in PTC via interacting with miR‐488‐3p.

Members of ADAM family are closely associated with a variety of biological events, like ectodomain shedding, cell proliferation, adhesion, migration, and invasion. ADAM9, as an important member of this family, is widely distributed in human tissues and involved in various biological processes.^36^, ^37^ ADAM9 is highly expressed in multiple cancers and is related to aggressive tumor phenotypes and poor clinical outcomes.^36^ ADAM9 has been found to be responsible for the growth and metastasis of thyroid cancer.^27^ We found that ADAM9 expression was higher in PTC tissues and cells than their controls. ADAM9 was demonstrated to be a target of miR‐488‐3p in non‐small cell lung cancer.^26^ We also confirmed that miR‐488‐3p could regulate ADAM9 expression in PTC cells. Therefore, we further determined the association between CASC9 and ADAM9. Our results showed that ADAM9 expression was positively related to CASC9 in human PTC tissues. An RIP assay with anti‐Ago2 antibody and expression analysis demonstrated that CASC9 acted as a ceRNA for miR‐488‐3p to elevate ADAM9 expression. We also found overexpression of ADAM9 partially reversed the suppressed proliferation, migration, and invasion of PTC by CASC9 silencing. Additionally, this study found downregulation of CASC9 in mice notably increased miR‐488‐3p, but decreased ADAM9 expression in tumors. Although we did not further evaluate the regulatory mechanism among CASC9, miR‐488‐3p, and ADAM9 in vivo using restore experiments, considering the detailed regulatory mechanism among them has been verified in PTC cells, our results were sufficient to demonstrate that CASC9 regulated the malignant phenotypes of PTC via miR‐488‐3p/ADAM9. ADAM9 has been found to be an important regulator of EGFR‐Akt signaling, which is a crucial signal pathway in PTC^38^, ^39^, ^40^, ^41^; hence, we further analyzed the role of CASC9 on EGFR‐Akt signaling and the results showed that downregulation of CASC9 significantly decreased the activation of EGFR‐Akt signaling, the effect of which was reversed by anti‐miR‐483‐3p, but further strengthened by miR‐488‐3p mimic in PTC cells. In general, these results suggested that CASC9 promoted the malignant properties in PTC by sponging miR‐488‐3p to relieve its inhibition on ADAM9 expression, leading to the activation of EGFR‐Akt signaling.

In conclusion, our study proved for the first time that elevated CASC9 expression promoted the proliferation and metastasis of PTC. The data described a novel mechanism of CASC9 in cancers. CASC9 facilitated the aggressive phenotypes of PTC by regulating miR‐488‐3p/ADAM9 pathway. This study will increase our understanding of the progression of PTC and may provide a novel target for the treatment of this disease.

## CONFLICT OF INTEREST

The authors have no conflict of interest.
